The article "NILCO biomarkers in breast cancer from Chinese patients" was published in 2014. Journal: BMC Cancer.

# NILCO biomarkers in breast cancer from Chinese patients

**DOI:** 10.1186/1471-2407-14-249

**Published:** 2014-04-09

**Authors:** Laronna S Colbert, Kaamilah Wilson, Sungjin Kim, Yuan Liu, Gabriela Oprea-Ilies, Corey Gillespie, Toi Dickson, Gale Newman, Ruben Rene Gonzalez-Perez

**Affiliations:** 1 Hematology/Oncology Section, Morehouse School of Medicine, Atlanta, GA 30310, USA; 2 Current address: Department of Hematology/Oncology, Atlanta Veterans Affairs Medical Center, Decatur, GA 30033, USA; 3 Department of Microbiology, Biochemistry and Immunology, Morehouse School of Medicine, Atlanta, GA 30310, USA; 4 Department of Biostatistics & Bioinformatics, Winship Cancer Institute, Rollins School of Public Health, Emory University, Atlanta, GA 30322, USA; 5 Department of Pathology and Laboratory Medicine, Grady Campus, Emory University, Atlanta, GA 30032, USA

## Abstract

**Background:**

Notch, IL-1 and leptin are known pro-angiogenic factors linked to breast cancer development, tumor aggressiveness and poor prognosis. A complex crosstalk between these molecules (NILCO) has been reported in breast cancer cell lines. However, whether NILCO biomarkers are differentially expressed in estrogen responsive (ER+), unresponsive (ER-) and triple negative (TNBC) breast cancer tissues is unknown.

**Methods:**

Expression levels of nine NILCO and targets [Notch1, Notch4, JAG1, DLL4, VEGF, VEGFR2 (FLK-1), leptin, leptin receptor (OB-R) and interleukin-1 receptor type I (IL-1R tI)] were examined via immunohistochemistry in breast cancer tissue microarrays from Chinese patients (ER+, n=33; ER-, n=21; TNBC, n=13) and non-malignant breast tissue (n=5; Pantomics, Inc.) using a semi-quantitative analysis of intensity staining, HSCORE.

**Results:**

Categorical expression of NILCO and targets (+ or -) was similar among all cancer tissues. However, TNBC showed differential localization pattern of NILCO. TNBC showed fewer nuclei and cytoplasms positive for Notch4 and JAG1, but more cytoplasms positive for leptin. In addition, fewer TNBC stromas were positive for Notch1 and Notch4, but 100% of TNBC stromas were positive for VEGFR2. Moreover, TNBC had lower DLL4 and IL-1R tI expression. TNBC and ER- showed higher expression of EGFR, but lower expression of AR. Leptin and OB-R were detected in more than 61% of samples. Leptin positively correlated to OB-R, JAG1, VEGF, and marginally to IL-1R tI. Notch1 positively correlated to IL-1R tI. EGFR and Ki67 were positively associated to Notch1, but no associations of NILCO and targets with p53 were found.

**Conclusions:**

Present data suggest that NILCO components are differentially expressed in breast cancer. TNBC showed distinctive patterns for NILCO expression and localization. The complex crosstalk between leptin, IL-1 and Notch could differentially drive breast cancer growth and angiogenesis. Furthermore, the analysis of NILCO and targets using Pathway Studio9 software (Ariadine Genomics) showed multiple molecular relationships that suggest NILCO has potential prognostic biomarker value in breast cancer.

The article "NILCO biomarkers in breast cancer from Chinese patients" was published in 2014. Journal: BMC Cancer.

## Background

Breast cancer is a heterogeneous disease with four major genetic-signature subtypes [1]. However, breast cancer can be broadly divided into two main groups: 1) Estrogen receptor positive (ER+) and triple negative breast cancer (TNBC: ER-, PR- and HER2-). The majority of breast cancers are ER+, respond to estrogens, and are commonly treated with anti-hormonal and HER2 (ErbB-2) targeted therapies. ER+ positive and HER2/neu+ breast cancer cells show suppressed Notch signaling, which is probably limited by the overwhelming proliferative and survival effects of ER and HER2-dependent pathways [2].

In contrast, TNBC is mostly dependent on growth factors [*i.e*., insulin, insulin-like growth factor-I (IGF-I) and adipokines] [3,4]. This aggressive form of the disease accounts for 15% of all invasive breast cancers showing an acutely early onset. TNBC is associated with poor survival and resistance to common therapeutic treatments. This difficult-to-treat form of breast cancer shows a tendency to overcome drug effectiveness [5].

Notch signaling is a hallmark of breast cancer [6,7]. The role of Notch in breast cancer development has long been studied, particularly relative to its effects on angiogenesis [8]. Notch expression correlates to poor prognosis and drug resistance of breast cancer patients [9,10]. A particular feature of Notch signaling is its variable outcomes, which are dependent on cell and microenvironment types [7]. Ductal and lobular breast carcinomas show variable levels of Notch expression [2].

Notch signaling is a key mediator of proliferation, survival, and possibly malignant invasion of TNBC. These data suggest that TNBC is heavily dependent on Notch signaling [11]. In line with this notion, TNBC seems to differentially-activate Notch. Indeed, Notch1 and Notch4 are overexpressed in TNBC [12]. Moreover, in contrast to normal and ER+ breast cancer tissues, the activation of Notch in ER– breast cancer is linked to survivin upregulation (an apoptosis inhibitor and cell cycle regulator), which suggests ER- breast cancer cells are dependent on Notch-survivin signaling [13].

Recent data indicate that breast cancer development is likely related to lifestyle and the result of being overweight. Obesity is associated with more than 100,000 incidents of cancer in the United States every year, particularly cancers of the breast, colon, and endometrium. The specific molecular mechanisms involved in the development of obesity-related breast cancers are unknown. However, the general picture suggests that obesity-related breast cancer is the consequence of multi-factorial causes [14,15]. Several molecules with altered patterns of expression in obesity are involved in breast cancer (*i.e*., insulin and IGF-1, and adipokines) [16]. Leptin, the major adipokine secreted by adipose tissue, is also produced by malignant cells, and linked to increased levels of Notch and survivin in breast cancer [17-19], and can affect tumor angiogenesis [20]. Leptin signaling can influence pro-angiogenic, inflammatory and mitogenic events in breast cancer [21-24].

The article "NILCO biomarkers in breast cancer from Chinese patients" was published in 2014. Journal: BMC Cancer.

We have previously unveiled a complex crosstalk between Notch, IL-1 and leptin (NILCO) in breast cancer cell lines, which could be essential for leptin-induced proliferation, inflammation and angiogenesis [17]. Moreover, a functional Notch-leptin axis is found in mouse carcinogenic-induced [18] and syngeneic breast cancer [19]. In these mouse models, leptin signaling induces both the expression and activation of Notch. However, it is unknown whether NILCO and its targets could correlate and/or are differentially-expressed in human TNBC, ER-, and ER+ breast cancer tissues.

We propose that specific associations between NILCO biomarkers occur in breast cancer, which may differ in TNBC. To this end, we examined the expression and cellular localization of NILCO, and targets, via immunohistochemistry in a commercial array of breast cancer biopsies from Chinese patients. Data were also analyzed *in silico* via Pathway Studio9 software (Ariadine Genomics, MD) [4]. Data analyses suggest that significant associations exist between NILCO and targets in breast cancer tissues. Higher levels of leptin and Notch1 were found in malignant compared to non-malignant tissues. TNBC showed lower levels of DLL4 and IL-1R tI compared to ER- and ER+ breast cancer. TNBC and their stromas showed differential cellular localization of Notch1, Notch4, JAG1, leptin and VEGFR2. Taken together, these results suggest that differential patterns of NILCO and targets are found in TNBC versus ER- and ER+ breast cancer. Present data support the idea for the potential use of NILCO and related molecules as biomarkers in breast cancer.

## Methods

### Reagents and antibodies

Polyclonal antibodies for Notch4, OB-R amino terminus, DLL4, IL-1 R tI, VEGF, VEGFR2, Jagged1 (JAG1) and leptin were obtained from Santa Cruz Biotechnology, Inc. (Santa Cruz, CA). Polyclonal anti-Notch2 and -Notch3 were from Abcam Inc. (Cambridge, MA). Monoclonal anti-Notch1 antibody and other chemicals were purchased from Sigma-Aldrich (St. Louis, MO). Vectastin ABC-APK and Vectamount were obtained from Vector Laboratories (Burlingame, CA). Hematoxilyn was purchased from Dako Corporation, Carpinteria, CA.

The article "NILCO biomarkers in breast cancer from Chinese patients" was published in 2014. Journal: BMC Cancer.

### Tissue microarray

Breast cancer tissue arrays from female Chinese were obtained from Pantomics, Inc. (Richmond, CA). Biopsies features included age, grading, TNM staging, and receptor status of estrogen (ER), androgen (AR), progesterone (PR), epidermal growth factor receptors (ErbB1/EGFR/HER1 and ErbB2/HER2)*,* and p53 and Ki67 expression data. However, no information on body weight of patients was available. Each slide contained 150 cores, including 75 cases in duplicate of normal/hyperplastic specimens (n=3), fibroadenomas (n=2), ductal carcinoma in situ (DCIS, n=2), Paget’s disease (n=1) and invasive carcinomas (ER^+^, n=33; ER^-^, n=21 and TNBC, n=13) showing diverse levels of PR and HER2 expression. The studies were focused on non-malignant (n=5) and invasive carcinoma samples (ER+, ER- and TNBC; n=67).

### Immunohistochemisty (IHC)

IHC staining was performed on 12 separate microarray slides. The following specific antibodies were used to analyze nine antigens: anti-Notch1, Notch4, DLL4, JAG1, leptin, leptin receptor (OB-R), VEGF, VEGFR2 (FLK-1) and IL-1R tI. Staining patterns of 1206 tissue samples were evaluated by two independent observers in a blind manner. Three slides were used for negative controls (no primary antibody) incubated with secondary antibodies (anti-rabbit; anti-mouse and anti-goat-HRP, respectively; Vector Lab.).

### HSCORE determination

Staining intensity of cells in tissue arrays was evaluated as negative or positive in three different bright fields (≥100 cells/field). Semi-quantitative HSCORE was calculated for each antigen using the following equation: HSCORE = ∑ pi(i +1), where “i” was the intensity with a value of 0, 1, 2, or 3 (negative, weak, moderate or strong, respectively) and “pi” was the percentage of stained cells for each intensity [25,26].

### *In silico* analysis of NILCO and targets interaction networks in breast cancer

Pathway Studio9 software (Elsevier, Ariadine Genomics, MD) was used to evaluate NILCO and its targets’ interactions in breast cancer tissue arrays. HSCORE of antigens showing significantly relationships in breast cancer were imported into the pathway software and analyzed.

### Statistics

HSCOREs for each antigen were determined twice, averaged, named A_HSCORE and used in the analyses. Pearson or Spearman correlation coefficients were used to compare the concordance between results from duplicate breast tissue samples and pairwise correlation between A_HSCOREs from the nine antigens analyzed in the microarray. The outcome was defined for three types of breast cancers according to the expression of ER, PR and HER2 (ER^+^, ER^-^and TNBC). Predictors were defined for A_HSCORE of nine antigens (continuous; 1–4) and dichotomized A_HSCORE (categorical: negative if HSCORE=1; positive otherwise). Covariate analyses were performed for p53, EGFR, Ki67, AR, grade, stage and age. The patients’ clinicopathological and histology characteristics, and the categorical and continuous A_HSCOREs were summarized for breast cancer and non-malignant disease patients. Univariate association between categorical HSCOREs and continuous A_HSCOREs for ER, PR, HER2, EGFR, AR, Ki67 and p53 expressions and grade and stage were compared by Chi-square or Fisher’s exact test. ANOVA (analysis of variance) was used to analyze age and Notch1 expression. Kruskal-Wallis test was also used to analyze continuous HSCOREs. All analyses were done using SAS 9.3 (SAS Institute, Inc.) with a significance level of 0.05.

The article "NILCO biomarkers in breast cancer from Chinese patients" was published in 2014. Journal: BMC Cancer.

## Results

### Breast cancer tissue arrays

The clinicopathological and histological characteristics of non-malignant and breast cancer patients are summarized in Table 1. Invasive breast adenocarcinomas were assigned to three main groups according their expression of ER, PR and HER2 (*i.e*., ER+, ER- and TNBC). Age, grade, stage, Ki67, and p53 expression statuses were well-balanced among breast cancer tissues in the three groups (ER+, ER- and TNBC). However, ER, PR, HER2, EGFR and AR statuses were significantly different among them.

**Table 1:** Clinicopathological and histology characteristics of breast cancer tissue microarray samples

	**Breast cancer**				**Non-malignant**
**Characteristic**	**ER- (n=21)**	**ER+(n=33)**	**TNBC (n=13)**	P-value*	**Hyperplasias (n=3) or Fibroadenomas (n=2)**
Age	50.86 (± 12.47)	48.67 (± 11.15)	48.69 (± 11.6)	0.778	34.2 (± 11.67)
Grade					
I	0 (0)	1 (3.03)	0 (0)	0.969	NA
II	6 (28.57)	10 (30.3)	3 (23.08)		
III	15 (71.43)	22 (66.67)	10 (76.92)		
Stage					
1	1 (4.76)	1 (3.03)	0 (0)	0.142	NA
2	17 (80.95)	20 (60.61)	5 (38.46)		
3	2 (9.52)	7 (21.21)	4 (30.77)		
4	1 (4.76)	5 (15.15)	4 (30.77)		
ER					
Negative	21 (100)	0 (0)	13 (100)	**<.001**	2 (40)
Positive	0 (0)	33 (100)	0 (0)		3 (60)
PR					
Negative	19 (90.48)	11 (33.33)	13 (100)	**<.001**	2 (40)
Positive	2 (9.52)	22 (66.67)	0 (0)		3 (60)
HER2					
Negative	2 (9.52)	12 (36.36)	13 (100)	**<.001**	5 (100)
Positive	19 (90.48)	21 (63.64)	0 (0)		NA
EGFR					
Negative	13 (61.9)	31 (93.94)	8 (61.54)	**0.004**	5 (100)
Positive	8 (38.1)	2 (6.06)	5 (38.46)		NA
AR					
Negative	14 (66.67)	13 (39.39)	13 (100)	**<.001**	3 (60)
Positive	7 (33.33)	20 (60.61)	0 (0)		2 (40)
Ki67					
Negative	8 (38.1)	10 (30.3)	5 (38.46)	0.791	5 (100)
Positive	13 (61.9)	23 (69.7)	8 (61.54)		NA
P53					
Negative	16 (76.19)	24 (72.73)	9 (69.23)	0.903	5 (100)
Positive	5 (23.81)	9 (27.27)	4 (30.77)		NA

Data are presented as number of patients (%) or mean (± SD). ER: estrogen receptor; TNBC: triple negative breast cancer; PR: progesterone receptor; HER2: human epidermal growth factor receptor type 2; EGFR: epidermal growth factor receptor 1; AR: androgen receptor; Ki67: a proliferation marker; p53: a tumor suppressor protein. *The p-value is calculated by ANOVA for age and chi-square test or Fisher’s exact test for other covariates, where appropriate. Numbers in ”bold” show significant differences.

The article "NILCO biomarkers in breast cancer from Chinese patients" was published in 2014. Journal: BMC Cancer.

The majority of TNBC were grade III and stage III invasive ductal carcinomas. ER+ and ER- breast cancers were mainly invasive ductal carcinomas grade III and stage II (see Table 1). Approximately one third of TNBC and ER- breast cancers were positive for EGFR1. Notably, ER+ breast cancers were negative for EGFR1. Additionally, p53 expression was low in all breast cancers. In contrast, more than 50% of breast cancer samples were positive for Ki67 proliferation marker, which differed from non-malignant tissues (Table 1).

### Detection of NILCO and targets in breast cancer tissue arrays

Figure 1 shows representative images of staining of the nine antigens detected in invasive breast carcinomas [n=67; TNBC (n=13; 19%) and ER+(n=33; 49%) and ER- breast cancers (n=21; 31%)] and non-malignant breast tissues (n=5). Other breast cancer types were not included. NILCO and targets were detected in invasive breast adenocarcinomas and non-malignant breast tissues. Majority of breast cancers were positive for Notch1, DLL4 and VEGF.

**Figure 1:** **Immunohistochemical (IHC) detection of NILCO and targets in tissue arrays from breast cancer and non-malignant patients.** Representative pictures of immunohistochemical staining from breast cancer TNBC **(A)**, ER+ **(B)**, ER- **(C)** and non-malignant tissues **(D)** and, IHC negative controls **(E)** for the expression of NILCO and targets. Arrows show positive staining of NILCO components: Notch1 **(a)**, Notch4 **(b)**, DLL4 **(c)**, JAG1 **(d)**, leptin **(e)**, OB-R **(f)**, IL-1R tI **(g)** and targets VEGF **(h)** and VEGFR2 **(i)**, respectively. No staining was found in IHC-negative controls using anti-mouse **(j)**, anti-rabbit **(k)** and anti-goat **(l)** secondary antibodies. Magnification ×10.

Continuous A_HSCORE (positive or negative) of Notch1, Notch4, JAG1, OB-R, VEGF and, VEGFR2 were not significantly different among breast cancers irrespective of their expression of ER, HER2 and PR. Notch1, DLL-4 and, VEGF were detected in most malignant tissues. Leptin, OB-R, Notch4, JAG1 and, IL-1R tI were detected in more than 60% of breast cancer (ER+, ER- and, TNBC). In contrast, approximately 30% of these breast cancers showed immunoreactivity for VEGFR2. Leptin, OB-R, Notch1 and VEGFR2 were significantly lower in non-malignant tissues.

The article "NILCO biomarkers in breast cancer from Chinese patients" was published in 2014. Journal: BMC Cancer.

Remarkably, cellular localization of NILCO and targets was significantly different in TNBC compared to ER- and ER+ breast cancer (Table 2). A lower number of TNBC showed nuclear and cytoplasmatic staining for Notch4 and JAG1, but more TNBC cells showed cytoplasmatic staining for leptin. Additionally, VEGFR2 was mainly found in TNBC stromas, but fewer showed Notch1 and Notch4 staining (Table 2).

**Table 2:** Cellular localization of NILCO and targets within TNBC, ER+ and ER- breast cancer tissues

**Antigen**	**ER- (n=21)**	**ER+ (n=33)**	**TNBC (n=13)**	P-value*
**Notch1**	% positive	% positive	% positive	
Nucleus	90	97	83	0.0661
Cytoplasm	90	97	92	0.2480
Stroma	100	100	67	**<.001**
**Notch4**				
Nucleus	74	74	42	**0.0151**
Cytoplasm	90	77	50	0.0762
Stroma	100	100	67	**<.001**
**JAG1**				
Nucleus	84	77	50	**0.0281**
Cytoplasm	90	88	75	0.0694
Stroma	100	100	100	-
**DLL4**				
Nucleus	90	88	100	0.098
Cytoplasm	90	88	100	0.098
Stroma	0	0	0	-
**Leptin**				
Cytoplasm	68	65	100	**<.001**
Stroma	68	59	67	0.4055
**OB-R**				
Cytoplasm	84	71	67	0.3023
Stroma	84	79	83	0.3311
**IL-1R tI**				
Cytoplasm	90	97	83	0.3867
Stroma	100	100	83	0.2736
**VEGF**				
Nucleus	58	94	92	0.4221
Cytoplasm	100	91	92	0.4414
Stroma	91	100	100	-
**VEGFR2**				
Nucleus	84	85	50	0.0901
Cytoplasm	90	85	75	0.2668
Stroma	32	35	100	**<.001**

Staining for NILCO and targets within cancer (nucleus and cytoplasm) and tumor stroma is expressed as % of positive immunoreactivy in each group of breast cancer. ER: estrogen receptor; TNBC: triple negative breast cancer; Notch1 and 4: Notch receptor type 1 and 4; JAG1: Jagged1, a Notch ligand; DLL4: Delta like ligand 4, a Notch ligand; OB-R: leptin receptor; IL-1RtI: interleukin 1 receptor type I; VEGF: vascular endothelial growth factor; VEGFR2: vascular endothelial growth factor 2. *The p-value is calculated by ANOVA. Numbers in ”bold” show significant differences.

### Associations of HSCOREs of NILCO and targets with breast cancer type

Evaluation of A_HSCOREs showed diverse grade of expression of NILCO and targets in ER+, ER- and, TNBC (Table 3). A_HSCOREs of antigens in malignant and non-malignant tissues were used to calculate their univariate associations with breast cancer types.

**Table 3:** Univariate associations of A_HSCORE of NILCO and targets with TNBC, ER+and ER- breast cancer tissues

	**Breast cancer**				**Non-malignant**
**Antigen**	**ER- (n=21)**	**ER+ (n=33)**	**TNBC (n=13)**	P-value*	**Hyperplasias (n=3) or Fibroadenomas(n=2)**
**Notch1**	2.6 (2.01-3.19)	2.55 (1.9-3.19)	2.43 (1.68-3.18)	0.743	1.45 (1.04-1.86)
Negative	0 (0)	0 (0)	1 (7.69)	0.194	NA
Positive	21 (100)	33 (100)	12 (92.31)		5 (100)
**Notch4**	1.67 (1–3.48)	1.62 (1–2.9)	1.36 (1–2.87)	0.449	2 (1.23 - 2)
Negative	5 (25)	5 (16.13)	5 (41.67)	0.204	NA
Positive	15 (75)	26 (83.87)	7 (58.33)		3 (100)
**JAG1**	1.23 (1–2.09)	1.37 (1–3)	1.23 (1–2.24)	0.776	1.28 (1.11 - 2.28)
Negative	6 (28.57)	9 (27.27)	4 (30.77)	0.972	NA
Positive	15 (71.43)	24 (72.73)	9 (69.23)		5 (100)
**DLL4**	3.16 (1.91 - 3.66)	3.21 (2–3.87)	2.85 (1.19 - 3.36)	**0.028**	3.18 (2.59 - 3.68)
Negative	NA	NA	NA	NA	NA
Positive	21 (100)	33 (100)	13 (100)		5 (100)
**Leptin**	2.69 (1–4)	3.16 (1–4)	1.5 (1–3.84)	0.675	1 (1–1.24)
Negative	6 (28.57)	10 (30.3)	5 (38.46)	0.820	3 (60)
Positive	15 (71.43)	23 (69.7)	8 (61.54)		2 (40)
**OB-R**	1.06 (1–2.3)	1.11 (1–2.2)	1.05 (1–2.27)	0.924	1 (1–1.5)
Negative	7 (33.33)	10 (30.3)	5 (38.46)	0.867	4 (80)
Positive	14 (66.67)	23 (69.7)	8 (61.54)		1 (20)
**IL-1R tI**	3.65 (2.55 - 4)	3.72 (2.46 - 4)	3.31 (1–4)	**0.027**	3.99 (2.74 - 4)
Negative	7 (33.33)	10 (30.3)	5 (38.46)	0.194	NA
Positive	14 (66.67)	23 (69.7)	8 (61.54)		4 (100)
**VEGF**	3.74 (2.22 - 4)	3.67 (2.64 - 4)	3.77 (1.04 - 4)	0.767	3.96 (3.74 - 4)
Negative	NA	NA	NA	NA	NA
Positive	21 (100)	33 (100)	13 (100)		5 (100)
**VEGFR2**	1 (1–2)	1 (1–2)	1 (1–2)	0.506	1 (1–1.1)
Negative	15 (71.43)	20 (60.61)	9 (69.23)	0.685	3 (60)
Positive	6 (28.57)	13 (39.39)	4 (30.77)		2 (40)

Data are presented as median (range), and number of positive and negative tissues (%). ER: estrogen receptor; TNBC: triple negative breast cancer; Notch1 and 4: Notch receptor type 1 and 4; JAG1: Jagged1, a Notch ligand; DLL4: Delta like ligand 4, a Notch ligand; OB-R: leptin receptor; IL-1RtI: interleukin 1 receptor type I; VEGF: vascular endothelial growth factor; VEGFR2: vascular endothelial growth factor 2. Numbers in ”bold” show significant differences. *The p-value is calculated by ANOVA for Notch1 and Kruskal-Wallis test for the remaining numerical covariates; chi-square test or Fisher’s exact test for categorical covariates, where appropriate.

The article "NILCO biomarkers in breast cancer from Chinese patients" was published in 2014. Journal: BMC Cancer.

Expression of DLL4 and IL-1R tI were significantly different among the three breast cancer types (p=0.028 and 0.027, respectively; Table 3). Remarkably, TNBC showed the lowest levels of DLL4 and IL-1R tI.

### Correlations of NILCO and targets in breast cancer

Table 4 shows the pairwise analysis of continuous A_HSCOREs for the nine antigens in all invasive breast cancer tissues evaluated. Several correlations between NILCO and its targets were found in breast cancer tissue arrays. Positive detection of leptin within breast cancer tissues significantly correlated to higher levels of IL-1R tI, VEGF, and, OB-R. Additionally, OB-R was positively correlated to VEGF. Similarly, Notch ligands JAG1 and DLL4 positively correlated to leptin, OB-R, and, VEGF and OB-R expression, respectively. Furthermore, Notch receptors (Notch1 and Notch4) correlated to IL-1R tI and DLL4, respectively, whereas leptin was negatively correlated to VEGFR2.

**Table 4:** Pairwise correlation for NILCO in breast cancer tissue array

	**Notch1**								
**Notch1**	1.000	**Notch4**							
**Notch4**	0.132 (0.303)	1.000							
			**JAG1**						
**JAG1**	-0.128 (0.302)	-0.181 (0.155)	1.000						
				**DLL4**					
**DLL4**	-0.053 (0.672)	0.247 **(0.051)**	0.096 (0.441)	1.000					
					**Leptin**				
**Leptin**	0.055 (0.659)	-0.267 **(0.035)**	0.337 **(0.005)**	0.157 (0.206)	1.000				
						**OB-R**			
**OB-R**	0.098 (0.428)	0.026 (0.841)	0.288 **(0.018)**	0.228 (0.064)	0.359 **(0.002)**	1.000			
							**IL-1R tI**		
**IL-1R tI**	0.407 **(0.001)**	0.003 (0.985)	-0.024 (0.848)	0.087 (0.484)	0.221 (0.073)	0.153 (0.218)	1.000		
								**VEGF**	
**VEGF**	-0.137 (0.269)	-0.083 (0.517)	0.243 **(0.047)**	0.298 **(0.014)**	0.461 **(<.001)**	0.278 **(0.023)**	0.025 (0.844)	1.000	
									**VEGFR2**
**VEGFR2**	0.023 (0.852)	0.279 **(0.027)**	-0.132 (0.289)	0.057 (0.646)	-0.370 **(0.002)**	-0.001 (0.992)	0.044 (0.725)	-0.176 (0.154)	1.000

Data are presented as a Spearman correlation coefficient (p-value). Notch1 and 4: Notch receptor type 1 and 4; JAG1: Jagged1, a Notch ligand; DLL4: Delta like ligand 4, a Notch ligand; OB-R: leptin receptor; IL-1RtI: interleukin 1 receptor type I; VEGF: vascular endothelial growth factor; VEGFR2: vascular endothelial growth factor 2. *The p-value is calculated by ANOVA. Numbers in ”bold” show significant differences.

### Associations of A_HSCOREs of NILCO and targets with EGFR, AR, Ki67 and p53 expression

Table 5 shows the analysis of univariate associations of categorized and continuous A-HSCOREs of NILCO and targets in breast cancer tissue arrays with EGFR and AR expression. Notch1 expression was associated to EGFR1 expression (p=0.018; Table 5). However, the expression of EGFR1 was not significantly associated with the positive or negative detection (categorized A_HSCOREs) of NILCO or targets. DLL4, Notch1, IL-1R tI and VEGF were expressed in almost all breast cancer tissues irrespective of AR status (Table 5). In contrast, IL-1R tI expression was associated with AR expression (p=0.026; Table 5). All TNBC tissues analyzed were negative for AR.

The article "NILCO biomarkers in breast cancer from Chinese patients" was published in 2014. Journal: BMC Cancer.

**Table 5:** Univariate associations of HSCORE for NILCO and targets with EGFR and AR

	**EGFR**			**AR**		
**Antigen**	**Negative (N=52)**	**Positive (N=15)**	P-value*	**Negative (N=40)**	**Positive (N=27)**	P-value*
**Notch1**	2.44 (1.78- 3.06)	2.89 (2.28-3.50)	**0.018**	2.49 (1.84-3.09)	2.62 (1.99-3.25)	0.403
Negative	1 (1.92)	0 (0)	1.000	1 (2.5)	0 (0)	1.000
Positive	51 (98.08)	15 (100)		39 (97.5)	27 (100)	
**Notch4**	1.55 (1–3.48)	1.81 (1–2.5)	0.782	1.62 (1–3.48)	1.7 (1–2.5)	0.966
Negative	12 (25)	3 (20)	1.000	10 (27.03)	5 (19.23)	0.474
Positive	36 (75)	12 (80)		27 (72.97)	21 (80.77)	
**JAG1**	1.35 (1–3)	1.17 (1–2.09)	0.215	1.28 (1–2.43)	1.23 (1–3)	0.510
Negative	13 (25)	6 (40)	0.332	13 (32.5)	6 (22.22)	0.360
Positive	39 (75)	9 (60)		27 (67.5)	21 (77.78)	
**DLL4**	3.15 (1.91 - 3.87)	3.27 (1.19 - 3.66)	0.443	3.19 (1.19 - 3.65)	3.15 (2–3.87)	0.828
Negative	NA	NA	NA	NA	NA	NA
Positive	52 (100)	15 (100)		40 (100)	27 (100)	
**Leptin**	3.07 (1–4)	2.69 (1–4)	0.825	2.88 (1–4)	3.02 (1–4)	0.938
Negative	16 (30.77)	5 (33.33)	1.000	12 (30)	9 (33.33)	0.773
Positive	36 (69.23)	10 (66.67)		28 (70)	18 (66.67)	
**OB-R**	1.09 (1–2.3)	1.05 (1–1.26)	0.338	1.1 (1–2.27)	1.06 (1–2.3)	0.359
Negative	17 (32.69)	5 (33.33)	1.000	12 (30)	10 (37.04)	0.547
Positive	35 (67.31)	10 (66.67)		28 (70)	17 (62.96)	
**IL-1R tI**	3.67 (1–4)	3.52 (1.56 - 4)	0.255	3.53 (1–4)	3.86 (2.46 - 4)	**0.026**
Negative	1 (1.92)	0 (0)	1.000	1 (2.5)	0 (0)	1.000
Positive	51 (98.08)	15 (100)		39 (97.5)	27 (100)	
**VEGF**	3.64 (1.04 - 4)	3.81 (2.45 - 4)	0.625	3.67 (1.04 - 4)	3.74 (2.83 - 4)	0.635
Negative	NA	NA	NA	NA	NA	NA
Positive	52 (100)	15 (100)		40 (100)	27 (100)	
**VEGFR2**	1 (1–2)	1 (1–2)	0.957	1 (1–2)	1 (1–2)	0.757
Negative	34 (65.38)	10 (66.67)	0.927	27 (67.5)	17 (62.96)	0.701
Positive	18 (34.62)	5 (33.33)		13 (32.5)	10 (37.04)	

Data are presented as median (range), and number of positive and negative tissues (%). EGFR: epidermal growth factor receptor 1; AR: androgen receptor; Notch1 and 4: Notch receptor type 1 and 4; JAG1: Jagged1, a Notch ligand; DLL4: Delta like ligand 4, a Notch ligand; OB-R: leptin receptor; IL-1RtI: interleukin 1 receptor type I; VEGF: vascular endothelial growth factor; VEGFR2: vascular endothelial growth factor 2. * The p-value is calculated by ANOVA for Notch1 and Wilcoxon rank-sum test for the remaining numerical covariates; chi-square test or Fisher’s exact test for categorical covariates, where appropriate. Numbers in ”bold” show significant differences.

Table 6 shows the analysis of univariate associations of categorized and continuous A-HSCOREs of NILCO and targets in breast cancer tissue arrays with Ki67 and p53 expression. The analysis of univariate association of categorized and continuous A_HSCOREs of NILCO and targets showed that Notch1 and JAG1 expression were significantly higher in breast cancers positive for Ki67 (p=0.01 and p=0.004 respectively; Table 6). In contrast, continuous A_HSCORE of VEGF was marginally higher and negatively associated to Ki67 expression (p=0.056, Table 6). An inverse association of VEGFR2 with Ki67 positive staining was found in breast cancer tissue arrays (p=0.026, Table 6). Univariate association analysis of A_HSCOREs of NILCO and its targets did not show significant differences with p53 expression in breast tissue arrays (Table 6). Nevertheless, no differences in Ki67 or p53 reactivity were found among ER+, ER- and, TNBC (see Table 1).

The article "NILCO biomarkers in breast cancer from Chinese patients" was published in 2014. Journal: BMC Cancer.

**Table 6:** Univariate associations of HSCORE for NILCO and targets with Ki67 and p53

	**Ki67**			**p53**		
**Antigen**	**Negative (n=52)**	**Positive (n=15)**	P-value*	**Negative (n=40)**	**Positive (n=27)**	P-value*
**Notch1**	2.27(1.68-2.86)	2.69 (2.06-3.32)	**0.010**	2.51(1.82-3.20)	2.63 (2.13-3.13)	0.528
Negative	1 (4.35)	0 (0)	0.343	1 (2.04)	0 (0)	1.000
Positive	22 (95.65)	44 (100)		48 (97.96)	18 (100)	
**Notch4**	1.42 (1–2.82)	1.69 (1–3.48)	0.125	1.51 (1–3.48)	1.8 (1–2.87)	0.404
Negative	7 (33.33)	8 (19.05)	0.209	12 (26.67)	3 (16.67)	0.522
Positive	14 (66.67)	34 (80.95)		33 (73.33)	15 (83.33)	
**JAG1**	1.37 (1–2.24)	1.21 (1–3)	0.350	1.2 (1–3)	1.54 (1–2.43)	0.587
Negative	3 (13.04)	16 (36.36)	**0.044**	14 (28.57)	5 (27.78)	0.949
Positive	20 (86.96)	28 (63.64)		35 (71.43)	13 (72.22)	
**DLL4**	3.21 (1.91 - 3.66)	3.11 (1.19 - 3.87)	0.584	3.15 (1.19 - 3.66)	3.21 (2.59 - 3.87)	0.651
Negative	NA	NA	NA	NA	NA	NA
Positive	23 (100)	44 (100)		49 (100)	18 (100)	
**Leptin**	3.34 (1–4)	2.66 (1–4)	0.841	2.64 (1–4)	3.29 (1–4)	0.541
Negative	7 (30.43)	14 (31.82)	0.908	16 (32.65)	5 (27.78)	0.703
Positive	16 (69.57)	30 (68.18)		33 (67.35)	13 (72.22)	
**OB-R**	1.08 (1–2.27)	1.07 (1–2.3)	0.648	1.08 (1–2.3)	1.11 (1–2.2)	0.666
Negative	7 (30.43)	15 (34.09)	0.762	17 (34.69)	5 (27.78)	0.593
Positive	16 (69.57)	29 (65.91)		32 (65.31)	13 (72.22)	
**IL-1R tI**	3.63 (1–4)	3.63 (1.56 - 4)	0.714	3.65 (1–4)	3.55 (2.62 - 4)	0.847
Negative	1(4.35)	0 (0)	0.343	1 (2.04)	0 (0)	1.000
Positive	22(95.65)	44(100)		48(97.96)	18(100)	
**VEGF**	4(1.04 - 4)	3.56(2.22 - 4)	0.056	2.51(± 0.69)	2.63(± 0.5)	0.528
Negative	NA	NA	NA	1(2.04)	0(0)	1.000
Positive	23(100)	44(100)		48(97.96)	18(100)	
**VEGFR2**	1.09(1–2)	1(1–2)	**0.047**	1.51(1–3.48)	1.8(1–2.87)	0.404
Negative	11(47.83)	33(75)	**0.026**	12(26.67)	3(16.67)	0.522
Positive	12(52.17)	11(25)		33(73.33)	15 (83.33)	

Data are presented as median (range), and number of positive and negative tissues (%). Ki67: a proliferation marker; p53: a tumor suppressor protein; Notch receptor type 1 and 4; JAG1: Jagged1, a Notch ligand; DLL4: Delta like ligand 4, a Notch ligand; OB-R: leptin receptor; IL-1RtI: interleukin 1 receptor type I; VEGF: vascular endothelial growth factor; VEGFR2: vascular endothelial growth factor 2. *The p-value is calculated by ANOVA for Notch1 and Wilcoxon rank-sum test for the remaining numerical covariates; chi-square test or Fisher’s exact test for categorical covariates, where appropriate. Numbers in ”bold” show significant differences.

The article "NILCO biomarkers in breast cancer from Chinese patients" was published in 2014. Journal: BMC Cancer.

### Pathway studio analyses

*In silico* analysis of relationships between NILCO and its targets were performed using Pathway Studio9 software. Analysis of data published on expression of Notch, leptin, OB-R, IL-1R tI, and VEGF/VEGFR2 in breast cancer showed several correlations with tumor progression/angiogenesis. The software identified 1626 references reporting 160 connectivity hits that include regulation, biomarker, quantitative, and state changes (Figure 2). Further, analysis of EGFR, AR, Ki67, Notch, leptin, IL-1, VEGF and VEGFR2 genes showed their involvement in the regulation of Notch1, leptin, JAG1, and VEGF in carcinogenesis (1064 references; see Additional file 1).

**Figure 2:** **Processes and outcomes involving leptin, OB-R, Notch1, Notch4, IL-1R tI, JAG1, DLL4, VEGF, VEGFR2 (KDR), EGFR, AR and Ki67 (MKi67 gene) in the development of breast neoplasms.** Breast cancers showed a quantitative increase in the expression of leptin, OB-R, Notch1, Notch4, DLL4, JAG1, IL-1R tI, VEGF, VEGFR2, EGFR, AR and Ki67. Increased expression of leptin, Notch1, Notch4, JAG1, and VEGF upregulated the development of breast neoplasms. Elevated levels of leptin, OB-R, Notch1, DLL4, VEGF, AR, EGFR and Ki67 proteins are reported to be biomarkers for breast cancers (data obtained from 1064 references; see Additional file 1; Pathway Studio9, Ariadine Genomics).

## Discussion

Notch signaling is a hallmark of breast cancer that is frequently identified as an indicator of poor prognosis and advanced disease. Therefore, Notch signaling is being targeted for breast cancer treatment [7,27]. Additionally, increased leptin signaling has also been related to breast cancer growth, angiogenesis and poor outcomes [24]. Leptin increased the expression and activation of several members of the Notch family of proteins in breast cancer cells and derived tumors [17-19]. VEGF and VEGFR2 can be regulated by leptin-Notch crosstalk, which was also affected by IL-1 signaling. Therefore, Notch, IL-1 and leptin crosstalk outcome (NILCO) could be essential for the integration of leptin’s proangiogenic, pro-inflammatory and proliferative actions in breast cancer [17]. Leptin could also be involved in the development of drug resistance, metastasis and relapse of breast cancer, which are related to cancer stem cells [24,28]. Furthermore, leptin transactivated and induced the expression of ER [29], EGFR [30], HER2 [31,32] and IGF-1R [33] in breast cancer.

The article "NILCO biomarkers in breast cancer from Chinese patients" was published in 2014. Journal: BMC Cancer.

The abrogation of leptin signaling impaired the growth of tumors and expression of angiogenic biomarkers in human breast cancer xenografts [34,35], and in mouse carcinogenic-induced [18] and syngeneic mammary tumors, which was more evident in obese contexts [19,21]. Moreover, accumulated evidence from these pre-clinical studies in mice reinforces the idea that leptin-Notch crosstalk plays an important role in breast cancer. Nevertheless, whether NILCO and targets are differentially-expressed in human breast cancer tissues, in relation to ER, PR and HER2 as well as EGFR and AR statuses, is unknown.

Here we show that NILCO components (Notch1, Notch4, JAG1, DLL4, leptin, OB-R, IL-1R tI) and target molecules (VEGF and VEGFR2) were co-expressed in breast cancer tissues, irrespective of ER, PR and, HER2 statuses. Remarkably, TNBC shows a differential pattern of expression and cellular localization of NILCO. TNBC showed lower protein levels of IL-1R tI and DLL4, and fewer nuclei and cytoplasms were positive for Notch4 and JAG1. In contrast, more TNBC cytoplasms were positive for leptin. Moreover, TNBC stromas showed distinctive patterns of Notch1 and VEGFR2 immnoreactivities. Notch1 and Notch4 expression were lower, but VEGFR2 expression was higher in stromas from TNBC compared with ER- and ER+ breast cancer stromas.

Notch1 was found in the majority of breast cancer tissues evaluated. This data was in agreement with a previous report that showed 100% of Notch1 expression in TNBC [36]. Notch4 expression was previously found in 73% of TNBC cases (n=29) [36]. Present data show that fewer TNBCs were positive for Notch4 (58%) compared to ER- (75%) and ER+ (84%), but the differences were not significant. However, nuclear localization of Notch4 was significantly lower in TNBC malignant cells and stroma.

Present data further confirm previous findings showing that TNBC cells in culture (MDA-MB231) secreted more leptin (approximately four-fold) than ER+ breast cancer cells (MCF-7) [34]. Notch-induced transcriptional activity was not previously correlated with Notch receptor levels in breast cancer cell cultures, but Notch-induced gene transcription was highest in TNBC cells [2]. The global biological relevance of these findings is unclear. Nevertheless, present findings might indicate that TNBC could greatly depend on leptin’s actions, which could underline the role of NILCO in this breast cancer type.

The article "NILCO biomarkers in breast cancer from Chinese patients" was published in 2014. Journal: BMC Cancer.

Notch1 expression was also associated with the cell proliferation marker, Ki67. This marker was detected in approximately 60% of breast cancer independently of the expression of hormone receptors. It was previously reported that Ki67 is found in 90% of TNBC [12] and its expression correlates to Notch4, which is induced by Notch1 in breast cancer samples [2].

The transformation of normal breast epithelial cells by increased Notch signaling was previously linked to the repression of apoptosis *in vitro*[9]. Notch NICD1 interacted and mediated p53 inactivation through phosphorylation *in vitro*[37]. Additionally, it was also suggested that Notch signaling regulated apoptosis specifically caused by p53-induced expression of Puma and Noxa *in vitro*[6]. However, our present data suggest that p53 was not associated with the expression of NILCO and its targets, and is independent of hormonal receptor status. This data may also suggest that Notch-induced apoptosis in breast cancer *in vivo* may not always be p53 dependent.

TNBC and ER- breast cancers are not responsive to steroid hormones, but are highly aggressive tumors that respond to several other growth factor-related signals [5]. TNBC frequently show EGFR expression and resistance to EGFR drugs that could be driven by the Notch pathway [38]. In these cancers, Notch, leptin and OB-R could further contribute to tumor growth via increased the survival of breast cancer stem cells [24]. Indeed, the abrogation of Notch can negatively affect stem cells [10,27]. Moreover, inhibition of OB-R significantly reduces the expression of several stem cell self-renewal transcription factors (NANOG, SOX2, and OCT4), and induces a mesenchymal-to-epithelial transition in TNBC cells [39]. Our present investigations show that EGFR expression was found in more ER- and TNBC (five-fold) than ER+ tumors. Additionally, EGFR was associated with higher expression of Notch1. Interestingly, leptin-induced activation of EGFR was suggested as a potential mechanism that promotes metastasis as well as invasion and, migration of breast cancer [33].

Obesity could affect breast carcinogenesis by autocrine and paracrine actions mediated by two major adipokines: leptin and adiponectin [24]. Obese breast cancer patients show poor prognosis, higher aggressiveness, and drug resistance [40-42]. Accumulated evidence suggests that obesity could induce Notch signaling. Indeed, an intact leptin-Notch axis could be involved in obesity-related breast cancer [18,19]. However, diverse factors from adipose and other organs could also influence breast carcinogenesis and tumor growth. Therefore, more investigations are necessary to understand obesity-related breast cancer causes and mechanisms [43,44]. All tissue samples used in this investigation were from Asiatic women (mean age of approximately 50 years). Obesity in China is currently a health problem. In 2002, the prevalence of obesity in China was relatively low (overweight prevalence at about 22.8% and for obesity, 7.1%) compared with Western countries, but the rapid increase in obesity is alarming [45]. Unfortunately, body weight and obesity data were not available for the breast cancer tissues used in this study.

The article "NILCO biomarkers in breast cancer from Chinese patients" was published in 2014. Journal: BMC Cancer.

## Conclusions

For the first time, we are reporting on a comprehensive data analysis on protein levels of NILCO and targets in three major groups of breast cancer: TNBC, ER-, and ER+. TNBC showed distinctive patterns of expression and localization of NILCO, which suggests these molecules may be useful as markers for disease progression and aggressiveness. It is known that inhibition of Notch [9] and leptin signaling [17,21,34,39] can revert the transformed phenotype of human breast cancer cell lines. Thus, treatments aimed to abrogate NILCO could provide the development of novel therapeutic interventions. More research is needed to establish the biomarker and potential therapeutic values of NILCO, and target expression in breast cancer, particularly in obese contexts.

## Abbreviations

OB-R: Leptin receptor; IL-1R tI: Interleukin 1 receptor type I; NILCO: Notch interleukin 1 leptin crosstalk outcome; EGFR: Epidermal growth factor receptor; NANOG: A homeobox protein and transcription factor; SOX2: Sex determining region Y-box 2 protein; OCT4: Octamer-binding transcription factor 4; IGF-1R: Insulin like growth factor receptor 1; ER: Estrogen receptor; AR: Androgen receptor; PR: Progesterone receptor; HER2: Epidermal growth factor receptor 2; DLL4: Delta like notch ligand 4; JAG1: Jagged 1 protein (a Notch ligand); VEGF: Vascular endothelial growth factor; VEGFR2: Vascular endothelial growth factor receptor 2 or KDR; TNBC: Triple negative breast cancer cells; HSCORE: A semi-quantitative analysis of intensity staining.

## Competing interests

The authors declare that they have no competing interests.

## Authors’ contributions

RRGP designed and wrote up the current study. LSC was involved in the study design, immunohistochemistry assays and HSCORE determinations of NILCO and targets. GN developed the *in silico* analysis of NILCO relationships using Pathway Studio9 Program and contributed to writing and editing the manuscript. KW, CG and TD developed immunohistochemistry assays and HSCORE determinations of NILCO, and targets. GO, performed immunohistochemical and pathological analyses of tissue samples. SK and YL performed the statistical analysis and interpretation of data. All authors read and approved the final manuscript.

The article "NILCO biomarkers in breast cancer from Chinese patients" was published in 2014. Journal: BMC Cancer.

## Pre-publication history

The pre-publication history for this paper can be accessed here:

http://www.biomedcentral.com/1471-2407/14/249/prepub

## Supplementary Material

Additional file 1 List of references reporting relationships between NILCO and its targets in breast cancer. Click here for file
